This article has been retracted.

# SRCIN1 Suppressed Osteosarcoma Cell Proliferation and Invasion

**DOI:** 10.1371/journal.pone.0155518

**Published:** 2016-08-11

**Authors:** Peng Wang, Hu Wang, Xiaotao Li, Ying Liu, Chengbin Zhao, Daling Zhu

**Affiliations:** 1 Department of Orthopedics, The Fourth Hospital of Harbin Medical University, Harbin, Heilongjiang, 150001, China; 2 Department of Orthopedics, First Affiliated Hospital of Shantou University Medical College, Shantou, 515041, Guangdong Province, China; 3 Department of Orthopedics, The First Affiliated Hospital of Jiamusi University, Jiamusi, Heilongjiang, 154000, China; 4 Clinical medicine Grade Four, Harbin Medical University, Harbin, Heilongjiang, 150001, China; 5 Department of Biopharmaceutical Sciences, College of Pharmacy, Harbin Medical University Daqing, Daqing, 163319, China; 6 Biopharmaceutical Key Laboratory of Heilongjiang Province, Harbin, 150081, China; University of South Alabama Mitchell Cancer Institute, UNITED STATES

## Abstract

SRCIN1 (SRC kinase signalling inhibitor 1) is a new tumor suppressor gene. Previous studies showed that SRCIN1 played a tumor suppressor role in the development of lung cancer and breast cancer. However, the role of SRCIN1 in osteosarcoma is still unknown. In this study, we demonstrated that SRCIN1 was downregulated in osteosarcoma cell lines compared with osteoblastic cell line. Moreover, SRCIN1 was downregulated in osteosarcoma tissues compared with the adjacent tissues. Further investigation revealed that overexpression of SRCIN1 inhibited the osteosarcoma cell line MG-63 proliferation. This effect was confirmed by measuring the ki-67 and PCNA expression. SRCIN1 overexpression promoted E-cadherin expression and suppressed N-cadherin, Vimentin and Snail expression, suggesting that SRCIN1 overexpression inhibited EMT of the osteosarcoma cell. In addition, ectopic expression of SRCIN1 inhibited the MG-63 cell colony formation and invasion. These data suggested that SRCIN1 acted as a tumor suppressor gene in the development of osteosarcoma.

## Introduction

Osteosarcoma is one of the most common primary bone malignancies in young adults and adolescents, with an estimated 5.6 per million children suffering from osteosarcoma yearly[1–4]. It occurs mostly in long extremity bone and around regions with active bone growth[5–8]. Despite the advances in treatment strategies of osteosarcoma, the 5-year survival rate of osteosarcoma patients is still poor[3, 9–12]. Thus, it is important to find the molecular mechanisms underlying the development of osteosarcoma and to identify novel biomarkers for the treatment, diagnosis and prognosis of this tumor[13–16].

SRCIN1 (SRC kinase signalling inhibitor 1), also named as p140 Cas-associated protein (p140CAP), contains two regions of highly charged amino acids, two proline-rich regions and two coiled-coil domains[17–20]. Previous studies demonstrated that SRCIN1 played an important role in Src inactivation and acted as a tumor suppressor gene in cancers[18, 21]. For example, Cao et al[22]. demonstrated that miR-150 acted as an oncogene through repressing SRCIN1 translation in lung cancer. Sharma et al[23]. showed that SRCIN1 inhibited tumor growth and impaired invasive properties of cancer cells by regulating the tyrosine kinase Src or E-cadherin/EGFR signaling pathways. In addition, the expression of SRCIN1 was inversely correlated with tumor malignancy in breast cancer. Damiano et al[18]. showed that SRCIN1 inhibited the highly metastatic breast carcinoma cells invasion by repressing cortactin-dependent cell motility. However, the role of SRCIN1 in osteosarcoma is still unknown.

In our study, we demonstrated that SRCIN1 was downregulated in the osteosarcoma cell lines and tissues. Overexpression of SRCIN1 inhibited the osteosarcoma cell proliferation and EMT. In addition, ectopic expression of SRCIN1 inhibited the MG-63 cell colony formation and invasion.

## Materials and Methods

### Clinical specimens and cell line cultured and transfection

Thirty osteosarcoma and adjacent nontumor bone tissues were collected from patients who underwent surgery in our hospital. Samples were immediately snap-frozen in liquid nitrogen. All of the patients have written informed consent to participate in this study. This study was approved by the Ethics Committee of The Fourth Hospital of Harbin Medical University and complied with the Declaration of Helsinki. Human osteosarcoma cell lines (U2OS, MG63, SAOS-2 and SOSP-9607) and one osteoblastic cell line (hFOB) were obtained from the ATCC (American Tissue Culture Collection). Lipofectamine 2000 (Dharmacon, TX, USA) was used to perform to cell transfection.

### RNA extraction and qRT-PCR

Total RNA from tissues and cells were isolated by using Trizol reagent (Invitrogen, Calsbad, CA, USA). Relative expression levels of SRCIN1 mRNA were measured by real-time PCR on the iQ5 Real-Time PCR Detection System (Bio-Rad, California, USA). Quantitative PCR primer for SRCIN1 was forward: 5’-AGCCCCGACAAAAGCAAAC-3’ and reverse: 5’-CCAAAGGAAGTCAATACAGGGATAG-3’; GAPDH was forward: 5’-AATGGGCAGCCGTTAGGAAA-3’ and reverse: 5’-TGAAGGGGTCATTGATGGCA-3’. GAPDH was used to as an endogenous control.

### Cell proliferation and colony formation

Cell Counting Kit-8 (CCK-8)(Dojindo; Kumamoto, Japan) was performed to measure the cell proliferation. Cells were cultured in 96-well plates for 1, 2or 3 days. The absorbance was detected at a wave length of 450 nm. For cell colony analysis, the cells were cultured at 1000cells/plate density and continue to seed for 2 weeks.

### Cell invasion

For cell invasion analysis, cells were seeded on the top side of transwell chambers coated with Matrigel (BD Bioscience). Mediumin the lower chambers containing 10% FBS acted as the chemo-attractant. After 24 h, the cells moving to the lower side of the membrane were fixed, stained with crystal violet and then counted by a microscope (BX51 Olympus, Japan).

### Western blot

Western blot analysis was measure according to previous studies. Proteins were isolated and detected using the BCA kit (Thermo Scientific, Rockford, IL). Proteins were separated by 10% SDS–PAGE and then transferred to PVDF membranes (Millipore, Danvers, MA). Membranes were cultured with primary antibodies GAPDH (Santa Cruz, CA) or SRCIN1 (Cell Signaling Technology). GAPDH was used as a loading control.

### Statistical analysis

Data was shown as means±SD. Statistics was measured using ANOVA or Student’s t-test using SPSS17.0. Statistical significance was shown asP<0.05.

## Results

### SRCIN1 was downregulated in the osteosarcoma cells

One representative patient was diagnosed as osteosarcomausing HE staining (Fig 1A). The mRNA expression of SRCIN1 was lower in the osteosarcoma cell lines (MG63, U2OS, SAOS-2 and HOS) than in the one osteoblastic cell line (hFOB) (Fig 1B). In line with this, the protein expression of SRCIN1 was lower in the osteosarcoma cell lines (MG63, U2OS, SAOS-2 and HOS) than in hFOB (Fig 1C).

**Fig 1:** The expression of SRCIN1 was downregulated in the osteosarcoma cells. (A) One representive patient was diagnosed as osteosarcoma using HE staining. (B) The mRNA expression of SRCIN1 was measured by using qRT-PCR. (C) The protein expression of SRCIN1 was measured by using western blot.

### SRCIN1 expression was reduced in the osteosarcoma tissues

SRCIN1 expression was also lower in the osteosarcoma tissues than in the adjacent nontumor tissues (Fig 2A). Meanwhile, SRCIN1 expression was downregulated in 29 patients (29/35, 82%) compared withthe adjacent tissues. We also confirmed that the protein expression of SRCIN1 was downregualted in the osteosarcoma tissues (Fig 2C).

**Fig 2:** SRCIN1 expression was reduced in the osteosarcoma tissues. (A) The mRNA expression of SRCIN1 was detected by using qRT-PCR in the osteosarcoma tissues and adjacent normal tissues. (B) SRCIN1 expression was downregulated in 29 patients (29/35, 82%) compared to the adjacent tissues. (C) The protein expression of SRCIN1 was measured by using western blot in the osteosarcoma tissues and adjacent normal tissues.

### SRCIN1 suppressed the osteosarcoma cell proliferation

As shown in Fig 3A and 3B, SRCIN1 expression was increased after transfected with SRCIN1 vector. Overexpression of SRCIN1 suppressed cell proliferation in the osteosarcoma cell line MG63 (Fig 3C). As shown in Fig 3D and 3E, the expression of ki-67 was decreased after transfected with SRCIN1 vector. Overexpression of SRCIN1 inhibited the PCNA expression in the MG-63 cell (Fig 3F and 3G).

**Fig 3:** SRCIN1 suppressed the osteosarcoma cell proliferation. (A) The protein expression of SRCIN1 was measured by using western blot in the MG-63 cells after treated SRCIN1 vector. (B) The mRNA expression of SRCIN1 was measured by using qRT-PCR in the MG-63 cells after treated SRCIN1 vector. (C) The cell proliferation was measured by CCK-8 analysis in the MG-63 cells. (D) The mRNA expression of ki-67 was measured by using qRT-PCR. (E) The protein expression of ki-67 was measured by using western blot in the MG-63 cells after treated SRCIN1 vector.(F) The mRNA expression of PCNA was measured by using qRT-PCR. (G) The protein expression of PCNA was measured by using western blot. *p<0.05, **p<0.01 and ***p<0.001.

### SRCIN1 inhibited epithelial–mesenchymal transition of the osteosarcoma cell

Overexpression of SRCIN1 enhanced E-cadherin mRNA expression while suppressed N-cadherin, Vimentin and Snail mRNA expression (Fig 4A). Moreover, we also showed that SRCIN1 overexpression promoted the expression of E-cadherin and inhibited the expression of N-cadherin, Vimentin and Snail (Fig 4B).

**Fig 4:** SRCIN1 inhibited epithelial–mesenchymal transition of the osteosarcoma cell. (A) The mRNA expression of E-cadherin, N-cadherin, Vimentin and Snail was measured by using qRT-PCR in the MG-63 cells after treated SRCIN1 vector. (B) The protein expression of E-cadherin, N-cadherin, Vimentin and Snail was detected by using western blot in the MG-63 cells after treated SRCIN1 vector.

### SRCIN1 repressed the osteosarcoma cell colony formation and invasion

Ectopic expression of SRCIN1 inhibited the MG-63 cell colony formation (Fig 5A). Moreover, overexpression of SRCIN1 suppressed the MG-63 cell invasion (Fig 5B).

**Fig 5:** SRCIN1 repressed the osteosarcoma cell colony formation and invasion. (A) Ectopic expression of SRCIN1 inhibited the MG-63 cell colony formation. (B) Overexpression of SRCIN1 suppressed the MG-63 cell invasion. ***p<0.001.

## Discussion

In this study, we demonstrated that SRCIN1 was downregulated in the osteosarcoma cell lines compared with osteoblastic cell line. Moreover, we showed that SRCIN1 expression was downregulated in osteosarcoma tissues compared with the adjacent tissues. Overexpression of SRCIN1 inhibited the osteosarcoma cell line MG63 proliferation. Furthermore, this effect was confirmed by measuring the ki-67 and PCNA expression. SRCIN1 overexpression promoted E-cadherin expression and suppressed N-cadherin, Vimentin and Snail expression. This result suggested that SRCIN1 overexpression inhibited EMT of the osteosarcoma cell. In addition, ectopic expression of SRCIN1 inhibited the MG-63 cell colony formation and invasion. These data suggested that SRCIN1 acts as a tumor suppressor gene in the development of osteosarcoma.

Previous studies showed that SRCIN1 actedas a crucial role in Src inactivation and acted as a tumor suppressor gene in a lot of tumors[18–21]. For example, Cao et al[22].showed that miR-150 acted as an oncogene by inhibiting SRCIN1 translation in lung cancer. Sharma et al[23]. demonstrated that SRCIN1 suppressed tumor growth and impaired invasive properties of cancer cells through inhibiting the tyrosine kinase Src or E-cadherin/EGFR signaling pathways. Moreover, the expression of SRCIN1 was inversely associated with tumor malignancy in breast cancer. Damiano et al[18]. demonstrated that SRCIN1 suppressed the highly metastatic breast carcinoma cells invasion by inhibiting cortactin-dependent cell motility. However, the role of SRCIN1 in osteosarcoma is still uncovered. In this study, we showed that SRCIN1 was downregulated in the osteosarcoma cell lines compared with osteoblastic cell line. Furthermore, we measured the SRCIN1 expression in 35 osteosarcoma patients’s tissues. We demonstrated that the expression of SRCIN1 was lower in the osteosarcoma tissues than in the adjacent non-tumor tissues. Meanwhile, SRCIN1 was downregulated in 29 patients (29/35, 82%) compared with the adjacent tissues.

We further investigated the role of SRCIN1 in osteosarcoma cell. Overexpression of SRCIN1 inhibited the osteosarcoma cell line MG63 proliferation. This effect was further confirmed by measuring the ki-67 and PCNA expression. SRCIN1 overexpression promoted the expression of E-cadherin while it suppressed N-cadherin, Vimentin and Snail expression. This result suggested that SRCIN1 overexpression inhibited EMT of the osteosarcoma cell. In addition, ectopic expression of SRCIN1 suppressed the MG-63 cell colony formation and invasion. These data suggested that SRCIN1 acted as a tumor suppressor gene in the development of osteosarcoma.

In conclusion, SRCIN1 may serve as a tumor suppressor gene in the development and metastasis of osteosarcoma. Given that ectopic expression of SRCIN1 suppresses cell proliferation and metastasis in the osteosarcoma, SRCIN1 may be a potent marker for the development of therapeutic strategies for patients with osteosarcoma.
